The article "PKMζ Inhibition Reverses Learning-Induced Increases in Hippocampal Synaptic Strength and Memory during Trace Eyeblink Conditioning" was published in 2010. Journal: PLoS One.

# PKMζ Inhibition Reverses Learning-Induced Increases in Hippocampal Synaptic Strength and Memory during Trace Eyeblink Conditioning

**DOI:** 10.1371/journal.pone.0010400

**Published:** 2010-04-29

**Authors:** Noelia Madroñal, Agnès Gruart, Todd C. Sacktor, José M. Delgado-García

**Affiliations:** 1 División de Neurociencias, Universidad Pablo de Olavide, Seville, Spain; 2 Departments of Physiology, Pharmacology, and Neurology, The Robert F. Furchgott Center for Neural & Behavioral Science, Downstate Medical Center, State University of New York, Brooklyn, New York, United States of America; Mount Sinai School of Medicine, United States of America

## Abstract

A leading candidate in the process of memory formation is hippocampal long-term potentiation (LTP), a persistent enhancement in synaptic strength evoked by the repetitive activation of excitatory synapses, either by experimental high-frequency stimulation (HFS) or, as recently shown, during actual learning. But are the molecular mechanisms for maintaining synaptic potentiation induced by HFS and by experience the same? Protein kinase Mzeta (PKMζ), an autonomously active atypical protein kinase C isoform, plays a key role in the maintenance of LTP induced by tetanic stimulation and the storage of long-term memory. To test whether the persistent action of PKMζ is necessary for the maintenance of synaptic potentiation induced after learning, the effects of ZIP (zeta inhibitory peptide), a PKMζ inhibitor, on eyeblink-conditioned mice were studied. PKMζ inhibition in the hippocampus disrupted both the correct retrieval of conditioned responses (CRs) and the experience-dependent persistent increase in synaptic strength observed at CA3-CA1 synapses. In addition, the effects of ZIP on the same associative test were examined when tetanic LTP was induced at the hippocampal CA3-CA1 synapse before conditioning. In this case, PKMζ inhibition both reversed tetanic LTP and prevented the expected LTP-mediated deleterious effects on eyeblink conditioning. Thus, PKMζ inhibition in the CA1 area is able to reverse both the expression of trace eyeblink conditioned memories and the underlying changes in CA3-CA1 synaptic strength, as well as the anterograde effects of LTP on associative learning.

## Introduction

Recently, two new lines of evidence have substantially strengthened the argument that the maintenance mechanism of LTP underlies the storage of memory [1]. First, activity-dependent changes in synaptic strength are induced at relevant brain sites during memory formation. In this regard, it has been shown that trace eyeblink conditioning and inhibitory avoidance both cause a detectable increase in synaptic transmission in the hippocampal CA1 area [2], [3]. Second, in the search for molecules that could be involved in both the maintenance of LTP and memory storage, a prime candidate termed protein kinase Mzeta (PKMζ) has recently appeared. PKMζ maintains the late, protein synthesis-dependent phase of LTP by increasing the number of functional AMPA receptors that are expressed at hippocampal synapses [4], [5]. Indeed, PKMζ is both necessary and sufficient for LTP maintenance [6]. In addressing these issues, a key tool has been ZIP, a selective, membrane-permeant peptide inhibitor of PKMζ that mimics the autoinhibitory regulatory domain of PKCζ that is missing from PKMζ [6]. ZIP reverses pre-established late-phase LTP when applied to hippocampal slices 1–5 h after LTP induction [7] and when injected in the hippocampus of anaesthetized rats 22 h after *in vivo* LTP induction [8]. That *in vivo* study also highlighted that PKMζ inhibition by ZIP in the hippocampus erases long-term memories encoded even weeks prior to the injection, a result reproduced in several other studies and other areas of the brain [9]–[11]. Thus a key question linking these two new lines of evidence that support the relationship between LTP and memory is whether PKMζ mediates the increase in synaptic strength induced by learning.

The article "PKMζ Inhibition Reverses Learning-Induced Increases in Hippocampal Synaptic Strength and Memory during Trace Eyeblink Conditioning" was published in 2010. Journal: PLoS One.

We therefore studied the effects of PKMζ inhibition by ZIP in the dorsal hippocampus on previously acquired trace eyeblink conditioning, a paradigm that, in humans, requires conscious knowledge [12] and/or declarative or explicit memory [13] of relevant relationships between conditioned (CS) and unconditioned (US) stimuli. We simultaneously examined the PKMζ inhibitor's effects on field EPSP (fEPSP) evoked at the CA3-CA1 synapse during the acquisition process [2]. CRs were determined from the electromyographic (EMG) activity of the orbicularis oculi muscle.

Because it was reported in a previous work that experimentally evoked LTP is able to occlude any further learning even for >10 days after potentiation disappearance [14], we also tested whether PKMζ inhibition reverses the effects of HFS-induced LTP before the eyeblink conditioning test. In both cases, we injected the standard dose of ZIP that locally reverses *in vivo* evoked LTP without affecting baseline synaptic transmission, and erases established memories [8], [11]. Results indicate that PKMζ inhibition in the hippocampus disrupts the retention of classically conditioned memories, using a trace paradigm, and the underlying experience-induced LTP, as well as reversing the deleterious effects of HFS-induced LTP on the acquisition of associative learning.

## Results

### Simultaneous recordings of orbicularis oculi EMG and hippocampal fEPSPs in cannula-implanted mice

Figure 1 illustrates the experimental design. The stability of both EMG and fEPSP recordings for >30 days in behaving mice has been reported previously [14]. Implanted electrodes in the upper lid allowed the generation of spontaneous eyeblinks and CRs without disrupting its kinematics. As illustrated in Figure 1C, CRs were easily distinguished in EMG records.

The article "PKMζ Inhibition Reverses Learning-Induced Increases in Hippocampal Synaptic Strength and Memory during Trace Eyeblink Conditioning" was published in 2010. Journal: PLoS One.

**Figure 1:** Experimental design and analysis of eyeblink data. (A) Animals were implanted with EMG recording electrodes in the orbicularis oculi (O.O.) muscle and with stimulating electrodes on the supraorbital nerve. For trace eyeblink conditioning, a tone was used as CS and an electric shock at the trigeminal nerve as US. The location of hippocampal stimulating (St.) and recording (Rec.) electrodes and of the injection cannula is illustrated in the top diagram. Abbreviations: DG, dentate gyrus; D, L, M, V, dorsal, lateral, medial, and ventral; Sch., Schaffer collaterals; Sub., subiculum. (B) Photomicrographs illustrating the location (white arrows) of the injection cannula and of the stimulating and recording sites. Calibration bar is 200 µm. (C) Schematic representation of the trace conditioning paradigm, illustrating CS and US stimuli, and the moment when a single electrical pulse (100 µs, square, biphasic) was presented to Schaffer collaterals (St. Hipp.). Examples of EMG and hippocampal extracellular records obtained from the 8th conditioning session of a representative animal are shown. Note the fEPSP evoked by the single pulse (St.) presented to Schaffer collaterals. (D) Three superimposed EMG traces recorded from the orbicularis oculi muscle of control animal following electrical stimulation (a single, 500-µs, cathodic pulse, 2 × threshold) of the supraorbital nerve. Note the characteristic R1 and R2 components of the evoked blink response [2]. (E) No significant differences (*P* = 0.575) in the latency to the R1 component between the three experimental groups were observed: controls (C), and ZIP- and scr-ZIP-injected mice. (F) Quantitative analysis of the area (expressed in µV × s) of the rectified EMG response corresponding to the R1 component of the evoked blink response. No significant differences (*P* = 0.302) between groups were observed. Drug infusions were carried out as indicated in the Methods section. Each bar in B and C represents the mean value collected from 3 animals ± s.e.m.

In Figure 1D is shown that reflexively evoked eyeblinks presented the characteristic R1 and R2 components, already described in different species of mammals, including mice [2]. Indeed, scr-ZIP and/or ZIP administration did not modify reflexively-evoked eyeblinks, as compared with controls (n = 3 animals per group). Indeed, the latency [F_(18,36)_ = 0.907; *P* = 0.575; Figure 1E] and the EMG amplitude [F_(18,36)_ = 1.213; *P* = 0.302; Figure 1F] of blinks evoked experimentally by the electrical stimulation of the ipsilateral supraorbital nerve presented no significant differences between groups.

The article "PKMζ Inhibition Reverses Learning-Induced Increases in Hippocampal Synaptic Strength and Memory during Trace Eyeblink Conditioning" was published in 2010. Journal: PLoS One.

The chronic implantation of stimulating and recording electrodes in the hippocampus allowed us to record the hippocampal extracellular activity and to follow the evolution of fEPSPs evoked in the CA1 area by the electrical stimulation of the ipsilateral Schaffer collateral/commissural pathway for >20 days (Figures 2A and 3A), despite the presence of an injection cannula also implanted in the CA1 area. The electrical stimulation of Schaffer collaterals disrupted the ongoing theta rhythm for only a brief (∼200 ms) period (Figure 1C). The actual location of hippocampal electrodes and cannula was checked at the end of each experiment (Figure 1B). We examined the putative effects of scr-ZIP and/or ZIP infusions on hippocampal EEG activities and on fEPSPs evoked at the CA3-CA1 synapse (n = 5 animals per group). As illustrated in Figures 2A and 2B, these two drugs did not modify the relative spectral power of theta, beta, and gamma bands [F_(2,8)_ = 0.218; *P* = 0.809] of EEG recordings collected from the hippocampal CA1 area. In addition, both input-output curves [F_(28,112)_ = 0.137; *P* = 0.874; Figure 2C] and paired-pulse tests [F_(10,40)_ = 0.298; *P* = 0.978; Figure 2D] evoked at the CA3-CA1 synapse did not indicate any significant difference in fEPSP slopes.

**Figure 2:** Effects on hippocampal EEG and on fEPSPs evoked at the CA3-CA1 synapse of ZIP and scr-ZIP injections in the CA1 area. (A) Examples of EEG recordings carried out in representative control (C), ZIP-, and scr-ZIP-injected animals. (B) Spectral power analysis of EEG recordings collected from the three experimental groups indicated no significant differences (*P* = 0.809). (C) Input/output curves of the CA3-CA1 synapse collected from the three experimental groups (n = 5 animals per group). No significant differences (*P* = 0.874) were observed in the data collected from the three groups. (D) Results collected from the paired-pulse test applied to the three groups of animals. No significant differences (*P* = 0.978) between groups were observed. Drug infusions were carried out as indicated in the Methods section. Each bar in B and each point in C and D represents the mean value collected from 5 animals ± s.e.m.

**Figure 3:** fEPSP and CR evolution for ZIP and scr-ZIP groups. (A, B) fEPSP slopes (A, white triangles) and percentage of CRs (B, white circles) for ZIP-injected animals (n = 10). For comparison, data (A, fEPSP, black triangles; B, percentage of CRs, black circles) corresponding to the scr-ZIP-injected group (n = 10) are also illustrated. In both groups, the injection took place 2 h before the 8th conditioning session (arrow). Illustrated fEPSP recordings (A, inset) were collected from the 1st and the 10th conditioning sessions of representative ZIP and scr-ZIP animals. Data are indicated as mean ± s.e.m. Asterisks indicate significant differences observed between the two groups for both fEPSP slopes (*P* = 0.021) and the percentage of CRs across training (*P* = 0.004) following ZIP injection.

The article "PKMζ Inhibition Reverses Learning-Induced Increases in Hippocampal Synaptic Strength and Memory during Trace Eyeblink Conditioning" was published in 2010. Journal: PLoS One.

### PKMζ inhibition reverses the normal acquisition of CRs

In order to determine whether the PKMζ inhibitor ZIP blocks classically conditioned established memories, we designed a first series of experiments in which two groups of animals (scr-ZIP and ZIP; n = 10 animals per group) were able to accomplish the two habituation sessions and the first 7 sessions of the classical conditioning test (Figure 3B). At this point, prior to drug injections, the percentage of CRs was 72.2±6.9% in the ZIP group and 79.8±6.9% in the scr-ZIP group, significantly larger than values collected during habituation sessions [F_(11)_ = 18.949; *P*<0.001], but with no significant differences between the two groups [F_(11,99)_ = 0.502; *P* = 0.898]. Two hours before the 8th conditioning session, animals were injected with either ZIP or scr-ZIP (Figure 3B, arrow). Following injections, the ZIP group presented a significantly lower percentage of CRs than those reached by the scr-ZIP group, from the 8th to the 10th conditioning sessions [F_(11,99)_ = 2.727; *P*<0.004].

The slope of fEPSPs evoked in both ZIP and scr-ZIP groups by single pulses presented to Schaffer collaterals during the CS-US interval increased steadily across conditioning sessions (Figure 3A), being significantly larger than baseline values for the 9th and 10th sessions [F_(11)_ = 2.428; *P* = 0.01] for the scr-ZIP group. In agreement with a previous description [2], [14], linear regression analyses applied to these fEPSP values demonstrated that they increased significantly across conditioning sessions (r = 0.89; *P* = 0.0007; slope  = 3.01) for the scr-ZIP control group. In contrast, the steady increase in fEPSP slopes evoked in the ZIP group was disrupted by ZIP injection (Figure 3A). Thus, fEPSP slopes collected from ZIP-injected animals were significantly lower than those recorded from the scr-ZIP group during the 9th and 10th conditioning sessions [F_(11,99)_ = 2.185; *P* = 0.021].

In summary, significant differences were observed between the two groups for both fEPSP slopes and the percentage of CRs following ZIP injection.

The article "PKMζ Inhibition Reverses Learning-Induced Increases in Hippocampal Synaptic Strength and Memory during Trace Eyeblink Conditioning" was published in 2010. Journal: PLoS One.

### PKMζ inhibition reverses LTP effects on associative learning

It has been reported that PKMζ inhibition by ZIP reverses established late-LTP [8], and that LTP induced before training sessions impairs spatial learning [15], place acquisition [16], and eyelid CRs [14]. Following these results, we decided to examine the effects on eyeblink conditioning of injecting scr-ZIP or ZIP in mice in which LTP was previously evoked (Figures 4A and 4B). LTP was evoked by the HFS protocol described in Methods. This HFS protocol was presented for 2 successive days (Figure 4A). After HFS, the same single stimulus used for baseline records was presented every 5 s for 15 min on the indicated days. In order to reverse LTP, animals (n = 10 per group) were infused in the hippocampus with scr-ZIP or ZIP 22 h after the 2nd HFS session. The following recording session took place 2 h after scr-ZIP or ZIP injection. As a result of peptide administration, the fEPSP slope was significantly smaller for the ZIP group than for the scr-ZIP (control) group during the 5 days following the injection [F_(9,81)_ = 2.331; *P* = 0.022; see Figure 4A]. HFS applied for 2 days in the scr-ZIP group evoked a well-defined LTP that remained above baseline values for at least 7 days [F_(9)_ = 21.622; *P*<0.001], even after the scr-ZIP injection. In contrast, fEPSP slopes for the ZIP group dropped from 167% (2nd HFS session) to baseline values immediately after ZIP injection. Although we did not examine a second pathway within these tetanized animals, ZIP had no significant effect on the CA3-CA1 synapse in the absence of a tetanic stimulation (Figure 2C). This point was checked in independent animals, and was consistent with previous results [8]. Thus, intrahippocampal injection of ZIP rapidly reversed the persistent potentiation of fEPSP slope, confirming and extending to awake animals previous *in vivo* work [8]. fEPSP slopes in ZIP-injected animals remained around baseline values until the end of the LTP-recording period, i.e., 7 days after ZIP injection.

**Figure 4:** LTP induction, fEPSP evolution, and learning curves for ZIP- and scr-ZIP-injected groups following two HFS sessions. (A, B) fEPSP slopes (A, white triangles) and percentage of CRs (B, white circles) for animals (n = 10) receiving HFS 9 and 8 days before the 1st habituation session (ZIP-injected group). Data (A, fEPSP, black triangles; B, percentage of CRs, black circles) corresponding to the scr-ZIP group (n = 10) are also illustrated. As a result of the LTP evoked by HFS, fEPSP slopes for the control group were significantly larger during the 5 days following injection (black arrow) than values collected from the ZIP group (A, *, *P* = 0.022). In contrast, the acquisition curve presented by the ZIP group was larger than that of controls (B, *, *P*<0.001). Differences in fEPSP slopes between ZIP and scr-ZIP groups were statistically significant from the 8th to the 10th conditioning sessions (A, *, *P*<0.05). Each point in A and B represents the mean value collected from 10 animals ± s.e.m. (C) Representative fEPSPs collected from the two groups, and corresponding to the LTP (1, 2) and conditioning (3, 4) periods as indicated in A. (D) Quantitative analysis of the linear relationships between fEPSP slopes and the percentage of CRs for the ZIP (top diagram, white circles) and the scr-ZIP (bottom diagram, black circles) groups across the 10 conditioning sessions. Each point represents the mean value collected from a single animal during the corresponding session. Regression lines are indicated when significant (*P*<0.05).

The article "PKMζ Inhibition Reverses Learning-Induced Increases in Hippocampal Synaptic Strength and Memory during Trace Eyeblink Conditioning" was published in 2010. Journal: PLoS One.

Seven days after scr-ZIP or ZIP injection, animals were subjected to the eyeblink conditioning paradigm described previously. Animals included in the scr-ZIP group were unable to present a normal learning curve, reaching a plateau of ∼35% of CRs from the 7th to the 10th conditioning sessions (Figure 4B). This unusual form of metaplasticity has been described in alert behaving mice using the same HFS protocol [14]. In contrast, the ZIP-injected group reached >65% of CRs from the 8th session on. The percentage of CRs obtained in the group previously injected with ZIP was larger than the corresponding values collected from the scr-ZIP group from the 2nd to the 10th conditioning sessions [F_(11,99)_ = 4.361; *P*<0.001]. Thus, PKMζ inhibition by ZIP was able to reverse the deleterious effects of inducing LTP before learning. Moreover, the slope of CA3-CA1 fEPSPs evoked in the ZIP group increased linearly (slope  = 3.01; r = 0.98; *P*<0.0001) across conditioning sessions, reaching ∼120% of baseline values from the 8th to the 10th conditioning sessions (Figures 4A and 4C). fEPSP slopes collected from the previously ZIP-injected animals during conditioning were significantly larger than baseline values from the 8th to the 10th conditioning sessions [F_(11)_ = 3.108; *P* = 0.001]. In contrast, fEPSPs recorded from the scr-ZIP group during the 10 conditioning sessions were not significantly different from baseline values (slope  = 0.74; r = 0.64; *P* = 0.09). Differences in fEPSP slopes between ZIP and scr-ZIP groups were statistically significant from the 8th to the 10th conditioning sessions [F_(11,99)_ = 1.575; *P*<0.05; Figure 4A].

As illustrated in Figure 4D, fEPSP slopes evoked in previously ZIP-injected mice were linearly related (r = 0.73; *P*<0.0001) to the percentage of CRs across conditioning sessions (slope  = 0.57), but were not for the scr-ZIP injected group (r = 0.17; *P* = 0.09).

The article "PKMζ Inhibition Reverses Learning-Induced Increases in Hippocampal Synaptic Strength and Memory during Trace Eyeblink Conditioning" was published in 2010. Journal: PLoS One.

As an additional control, and in order to check whether LTP can evoke permanent functional impairments of hippocampal circuits [2], [14] we carried out a complementary LTP study in 10 additional mice (Figure 5). To start, LTP was evoked by two successive HFS sessions as indicated above (Figure 4A). But, in this case, we induced a subsequent LTP after the first LTP has decayed to baseline values. LTP was evoked again by two additional HFS sessions presented on days 13 and 14 (Figure 5). In this situation, LTP was evoked with values slightly lower, but not significantly different [F_(24,96)_ = 3.950; *P* = 0.674], from those collected following the two prior HFS sessions. These results indicate that hippocampal circuits were still functionally active and not permanent damaged by the two earlier HFS sessions [see ref. 14 for details].

**Figure 5:** Characteristics of LTP evoked repetitively at the CA3-CA1 synapse. LTP was evoked in a group of control mice (n = 10) by the presentation of two successive HFS sessions. Evoked fEPSPs reached values significantly larger than baseline recordings for the indicated days [asterisk, *P*≤0.05; F_(24,96)_ = 3.950]. Subsequent HFS sessions were presented on days 13 and 14, i.e., after the first LTP has decayed to baseline values. Note that in this case, LTP was evoked again reaching values non-significantly different (*P* = 0.674) from those collected following the first two HFS sessions.

## Discussion

Inhibition of hippocampal PKMζ by ZIP, a cell-permeant peptide, blocks the development of a significant increase in hippocampal synaptic strength, disrupts retention of learned responses previously acquired with a trace conditioning test, a well-known paradigm that requires the participation of the hippocampus [2], [17], and reverses both the maintenance of tetanic LTP and its deleterious effects on the acquisition of conditioned eyeblink responses. In agreement with a previous report [8], ZIP did not seem to have any effect on on basal hippocampal synaptic transmission.

It has been reported that PKMζ maintains spatial, instrumental, and fear-motivated classically conditioned long-term memories, because injection of ZIP into the hippocampus or basolateral amygdala 22 h after learning causes a retrograde amnesia in all of these cases [8], [11]. Furthermore, ZIP is able to erase conditioned taste-aversion memory when infused into the insular cortex [9], [10]. Regarding trace eyeblink conditioning, if a persistent PKMζ activity in the hippocampus is necessary for the storage/recall of CRs, then inhibiting kinase activity at the end of conditioning training will cause the CS-US association to be forgotten. Present results indicate that, even after the associative test is learned, local ZIP injection into the hippocampus partially interferes with acquired memories and/or impairs the expression of CRs, disrupting its final asymptotic acquisition. In fact, ZIP administration was carried out at the conditioning session where maximal excitability changes in pyramidal CA3 and CA1 neurons have been reported during trace conditioning [18], [19] indicating that changes in excitability also contribute to the CR. In addition, there is no reason for proposing that ZIP in the hippocampus will be able to obliterate all established memories, because convincing studies have shown the involvement of specific neocortical regions in the storage of information initially processed in the hippocampus [20]. This is consistent with our observations that whereas the hippocampal experience-dependent increase in synaptic transmission was completely reversed by hippocampally-injected ZIP, the conditioned response was partially reversed.

The article "PKMζ Inhibition Reverses Learning-Induced Increases in Hippocampal Synaptic Strength and Memory during Trace Eyeblink Conditioning" was published in 2010. Journal: PLoS One.

As suggested by the present results, LTP induction not only modifies the expected synaptic response where the tetanization is aimed, but may also block the subsequent transfer of information toward other cortical circuits involved in associative learning [2], [14], [21], [22].

The presence of normal hippocampal EEG activities and CA3-CA1 synaptic transmission, after PKMζ inactivation by ZIP further confirms that ZIP has minimal effects on baseline synaptic responses [6]–[8], [23] and indicates that hippocampal circuits remain functionally unaffected after ZIP infusion.

Tetanus-induced LTP in the hippocampus is able to impair the acquisition of new conditioned behaviors, such as spatial learning when LTP is induced in the perforant pathway [15], [16], or trace eyeblink conditioning when LTP is induced at the CA3-CA1 synapse [2]. As reported recently [14], and further supported here, hippocampal LTP does not evoke permanent deficits in anterograde memories, but its effects remain for a certain (∼10 days) period. Here, PKMζ inactivation by intrahippocampal injection of ZIP 22 h after HFS rapidly reversed the induced LTP at the CA3-CA1 synapse, a finding also reported for the perforant pathway-dentate gyrus synapse [8]. ZIP injection also prevented the loss of anterograde memory acquisition caused by LTP induction in controls [14]. Thus, PKMζ not only maintains LTP at the CA3-CA1 synapse, but its inhibition speeds the process by which learning ability is recovered after LTP induction. LTP evoked in the present experiments can be considered a type 2 late-LTP [24], which is dependent on gene expression and protein synthesis [25].

The article "PKMζ Inhibition Reverses Learning-Induced Increases in Hippocampal Synaptic Strength and Memory during Trace Eyeblink Conditioning" was published in 2010. Journal: PLoS One.

It has been proposed that PKMζ acts by increasing the amount of GluR2-containing AMPA receptors at selected synapses, increasing in this way synaptic strength [4], [5]. But, since the potentiation declined spontaneously in control experiments (see Figure 4A, black triangles), we have to assume that the effects of PKMζ would have disappeared as well in the time elapsed from HFS to the beginning of the conditioning sessions (i.e., 10 days after the second HFS session). Therefore, it can be proposed that either hippocampal CA3-CA1 synapses remained potentiated in the controls, but not after ZIP infusion, or that ZIP/PKMζ interactions may be affecting other synaptic mechanisms, besides AMPA receptors.

The findings that the same local ZIP injection selectively reverses LTP and alters both associative memory and the underlying experience-dependent synaptic plasticity, indicates that the process that persistently alters synaptic networks involved in associative memory retention shares fundamental molecular properties with that of LTP maintenance. Thus the functional relationship between LTP and memory storage draws even closer.

## Materials and Methods

### Subjects

Experiments were carried out on C57Bl/6 male mice (3–5 months old; 25–35 g) obtained from an official supplier (University of Granada, Spain). A total of 40 successful (i.e., those from which a complete set of data was colleted, n = 10 per experimental group) animals were used in the present study. Mice were kept on a 12 h light/dark cycle with constant ambient temperature (21±1.5°C) and humidity (60±5%). Food and water were available *ad libitum*. Experiments were carried out in accordance with the guidelines of the European Union (2003/65/CE) for the use of laboratory animals in chronic experiments. Surgery and recording protocols were also approved by the Ethics Committee of Pablo de Olavide University (permit number CEEA-07/4).

### Surgery

Animals were anesthetized with 0.8–1.5% isoflurane, at a flow rate of 1–4 L/min oxygen, and implanted with stimulating electrodes on the left supraorbital nerve and with recording electrodes in the ipsilateral orbicularis oculi muscle (Figure 1A). Electrodes were made from 50 µm, Teflon-coated, annealed stainless steel wire (A-M Systems, Carlsborg, WA). Mice were also implanted with stimulating electrodes in the contralateral (right) Schaffer collateral/commissural pathway of the dorsal hippocampus (2 mm lateral and 1.5 mm posterior to bregma, and 1–1.5 mm from the brain surface [26]) and with a recording electrode placed in the right CA1 stratum radiatum (1.2 mm lateral and 2.2 mm posterior to bregma, and 1–1.5 mm from the brain surface). These hippocampal electrodes were made from 50 µm, Teflon-coated, tungsten wire (Advent Research, Eynsham, UK). A 25G stainless steel cannula was implanted close to the recording hippocampal electrode (1.6 mm lateral and 1.8 mm posterior to bregma, and 1 mm from the brain surface, i.e., 0.5 mm above the infusion target) and a bare silver wire affixed to the bone as ground. All the implanted wires were soldered to two four-pin sockets (RS Amidata, Madrid, Spain) and fixed to the skull with dental cement [2].

The article "PKMζ Inhibition Reverses Learning-Induced Increases in Hippocampal Synaptic Strength and Memory during Trace Eyeblink Conditioning" was published in 2010. Journal: PLoS One.

### Recording and stimulation procedures

For recordings, animals were placed in three separate small (5×5×10 cm) plastic chambers located inside a larger (25×25×40 cm) Faraday box. Both the EMG activity of the orbicularis oculi muscle and field EPSPs (fEPSPs) were recorded with Grass P511 differential amplifiers (Grass-Telefactor, West Warwick, RI).

### Intracranial drugs infusion

The chemicals used were the myristoylated peptide PKMζ inhibitor ZIP (10 nmol/1 µL saline; QCB and University Wisconsin Biotech peptide synthesis facility) and its corresponding scrambled control peptide, scr-ZIP, which comprises a random sequence of the same amino acids present in ZIP (10 nmol/1 µL saline; QCB). Injections of 1 µL of the ZIP or scr-ZIP solution, delivered at a rate of 0.2 µL/min, were made with a Hamilton syringe (2 µL) connected by a calibrated plastic tube to the implanted cannula. Drug injections took place 2 h before the selected recording session [8].

### Classical eyeblink conditioning

For trace conditioning, a tone (20 ms, 2.4 kHz, 85 dB) was presented as a CS, whilst the US consisted of a 500 µs, 3× threshold, square, cathodal pulse applied to the supraorbital nerve 500 ms after the end of the CS (Figure 1C). Animals received two habituation and 10 conditioning sessions. A conditioning session consisted of 60 CS-US presentations, and lasted ≈30 min. CS-US presentations were separated at random by 30±5 s. For habituation, only the CS was presented, also for 60 times per session, at intervals of 30±5 s. As criteria, we considered a “conditioned response” the presence, during the CS-US interval, of EMG activity lasting >20 ms and initiated >50 ms after CS onset. The integrated EMG activity recorded during the CS-US interval had to be at least 2.5 times greater than the averaged activity recorded immediately before CS presentation [see ref. 2].

During habituation and conditioning sessions, fEPSPs were evoked in the CA1 area by single 100 µs, square, biphasic pulses applied to Schaffer collaterals 300 ms after CS presentation. To avoid evoking a population spike, pulse intensity was set at 35–45% (0.05–0.15 mA) of the amount necessary to evoke a maximum fEPSP response [2], [27]. An additional criterion for selecting stimulus intensity was that a second stimulus, presented 40 ms later, evoked a larger (>20%) synaptic field potential than the first [28].

The article "PKMζ Inhibition Reverses Learning-Induced Increases in Hippocampal Synaptic Strength and Memory during Trace Eyeblink Conditioning" was published in 2010. Journal: PLoS One.

### Long-term potentiation

fEPSP baseline values (Figure 4A) were collected 15 min prior to LTP induction. For LTP induction, each animal was presented with two HFS sessions. Each HFS session consisted of five 200 Hz, 100 ms trains of pulses at a rate of 1/s. This protocol was presented six times, at intervals of 1 min. Thus, a total of 600 pulses were presented during an HFS session. The stimulus intensity during the HFS was set at the same value as that used for generating baseline recordings.

### Histology

At the end of the experiments, mice were deeply re-anesthetized (4% chloral hydrate solution, 10 mL/kg) and perfused transcardially with saline and 4% phosphate-buffered paraformaldehyde. Brains were dissected out, postfixed overnight at 4°C, and cryoprotected in 30% sucrose in PBS. Brain sections were obtained in a microtome (Leica, Wetzlar, Germany) at 50 µm. Selected dorsal hippocampus sections were mounted on glass slides and stained with 0.1% toluidine blue to determine the location of implanted cannula and electrodes (Figure 1B).

### Data storage and analysis

EMG and hippocampal extracellular activity, and 1-volt rectangular pulses corresponding to CS and US presentations, were stored digitally on a computer through an analog/digital converter (CED 1401 Plus, Cambridge, England). Data were analyzed off-line for quantification of CRs and fEPSPs with the Spike 2 (CED) program. Quantitative analysis of the area (expressed in µV × s) of the rectified EMG corresponding to the R1 component of the evoked blink response (Figure 1F) was analyzed as described elsewhere [29]. The spectral analysis of dominant frequencies present in the hippocampal field activity (Figure 2B) was carried out with the help following procedures described by Domingo et al. [30]. In short, the power spectrum of hippocampal extracellular activity collected during individual conditioning trials was computed, using the fast Fourier transform with a Hanning window, expressed as relative power and averaged across a complete session. This average was analyzed and compared using the wide-band model, considering the following bands: theta (4 to 9 Hz), beta (12 to 25 Hz), and gamma (25 to 100 Hz).

The slope of evoked fEPSPs was computed as the first derivative (volts/s) of fEPSP recordings (volts). Five successive fEPSPs were averaged, and the mean value of the slope during the rise-time period (i.e., the period of the slope between the initial 10% and the final 10% of the fEPSP) was determined. Computed results were processed for statistical analysis using the Sigma Stat for Windows package. Regression analyses were used to study the relationship between the fEPSP and the percentage of CRs. Data are always represented as the mean ± s.e.m. Acquired data were analyzed using a two-way ANOVA, with days as repeated measure and with a contrast analysis for a further study of significant differences.
